The article "A Breast Cancer Image Classification Algorithm with 2c Multiclass Support Vector Machine" was published in 2023. Journal: J Healthc Eng.

# A Breast Cancer Image Classification Algorithm with 2c Multiclass Support Vector Machine

**DOI:** 10.1155/2023/3875525

**Published:** 2023-07-08

**Authors:** Mohammed Abdul Wajeed, Shivam Tiwari, Rajat Gupta, Aamir Junaid Ahmad, Seema Agarwal, Sajjad Shaukat Jamal, Simon Karanja Hinga

**Affiliations:** ^1^Department of Computer Science and Engineering, Swami Vivekananda Institute of Technology, Secunderabad, Telangana, India; ^2^Department of Computer Science and Engineering, G L Bajaj Institute of Technology and Management, Greater Noida, Uttar Pradesh, India; ^3^Engineering and Technology, Career Point University, Kota, Rajasthan, India; ^4^Department of Computer Science and Engineering, Maulana Azad College of Engineering and Technology, Patna, India; ^5^SRM institute of Science and Technology, Delhi-NCR, Campus, Ghaziabad, India; ^6^Department of Mathematics College of Science, King Khalid University, Abha, Saudi Arabia; ^7^Department of Electrical and Electronic Engineering, Technical University of Mombasa, Mombasa, Kenya

## Abstract

Breast cancer is the most frequent type of cancer in women; however, early identification has reduced the mortality rate associated with the condition. Studies have demonstrated that the earlier this sickness is detected by mammography, the lower the death rate. Breast mammography is a critical technique in the early identification of breast cancer since it can detect abnormalities in the breast months or years before a patient is aware of the presence of such abnormalities. Mammography is a type of breast scanning used in medical imaging that involves using x-rays to image the breasts. It is a method that produces high-resolution digital pictures of the breasts known as mammography. Immediately following the capture of digital images and transmission of those images to a piece of high-tech digital mammography equipment, our radiologists evaluate the photos to establish the specific position and degree of the sickness in the breast. When compared to the many classifiers typically used in the literature, the suggested Multiclass Support Vector Machine (MSVM) approach produces promising results, according to the authors. This method may pave the way for developing more advanced statistical characteristics based on most cancer prognostic models shortly. It is demonstrated in this paper that the suggested 2C algorithm with MSVM outperforms a decision tree model in terms of accuracy, which follows prior findings. According to our findings, new screening mammography technologies can increase the accuracy and accessibility of screening mammography around the world.

## 1. Introduction

Breast cancer affects around one out of every 3,000 pregnant or breastfeeding women [1]. According to research, if a woman is diagnosed with breast cancer while pregnant, her odds of surviving are much lower than those of a no pregnant woman. According to the National Cancer Institute (NCI), about one in every ten women in the United States (US) will get breast cancer at some point in their lives [2]. In India, the overall incidence of breast cancer is lower than that in the United States, with 1 in 30 women being diagnosed with the disease. Breast cancer in men is extremely rare, accounting for only about 1% of all breast cancer cases in the United States [3]. Every year, approximately, 400 men die due to breast cancer. It is expected that African American males would die from breast cancer at a higher rate than white men in the future [4]. In 2014, statistics reveal that 40,000 women died and 232,670 new cases were identified in the United States of America. According to the most recent data from worldwide research, the number of breast cancer patients in India would grow from 1, 15,000 to 2, and 00,000 by the year 2030 [5].

The article "A Breast Cancer Image Classification Algorithm with 2c Multiclass Support Vector Machine" was published in 2023. Journal: J Healthc Eng.

Women are all affected by a sickness that leads to malignancy as a final outcome. Disease is a concern; if left untreated, the growth of dangerous cells results in slow damage and death as the cells multiply [6]. As a consequence of a genetic alteration that outgrows its control and becomes destructive as a result of changes in the deoxyribonucleic chemistry of the cell, unusual cells are generated [7]. It is important to remember that it does not cause damage to neighboring tissue while producing damage to a range of body capacities via the lymphatic system and evoking supplements from body tissues [8]. The most prevalent types of sickness include lymphoma, sarcoma, carcinoma, leukemia, and melanoma, to name a few. Carcinomas are the sort of illness that has been examined the most. Bosom cancer is a kind of cancer that affects mostly women and a few males all over the globe [9]. The pathologist's representation results in the anticipated tissue biopsy or fine needle yearning in the obsessive conclusion of bosom malignancy, as indicated by the pathologist. Breast cancer is distinguished from other types of cancer by the presence of abnormalities such as lumps and small calcifications [10]. In any case, irregularities are commonly ignored owing to the intricacy of the bosom structure, the low incidence of infection, and the fatigue of radiologists. It has been discovered that on any given day, 5,000 Malaysian women are diagnosed with breast cancer [11]. The majority of these women are between the ages of 30 and 60, with more than half of those afflicted being younger than the age of 50, according to Cancer Research. Radiologists have made the error of overlooking roughly 10 percent to 25 percent of unusual occurrences found during mammography [12]. Double reading is one method of reducing false-negative rates, which may increase location rates by 5 percent to 15 percent when they are not there. No matter how you look at it, double-time reading is both expensive and time-consuming [13]. Thus, researchers and radiologists are drawn to the issue of dealing with the bosom image for malignant growth discovery innovation because it is novel and interesting.

The article "A Breast Cancer Image Classification Algorithm with 2c Multiclass Support Vector Machine" was published in 2023. Journal: J Healthc Eng.

Both the left and right breasts are situated in the upper ventral region of a human body, on either side of the stem, and each breast encompasses a portion of the ventral region extending from the beginning of the second rib to the sixth rib, which contains the mammary gland [14]. The glandular tissue, fibrous tissue, fatty tissue, blood arteries, nerves, and ducts that make up the mature female breast are all present. The breast contains multiple lobes, generally 15 to 20, which are made up of lobules, which are a kind of lobule [15]. Alveoli and four lactiferous ducts make up this structure. During breastfeeding, the lactiferous ducts grow and create a tiny lactiferous sinus, which collects the milk produced by the body. Lactation occurs when milk escapes from the breast via a series of pores in the nipple [16]. The fibrous tissue covers the whole surface of the breast and connects the lobes of the breast together. It is located between the lobes of the gland and conceals its whole exterior except for the areola, which is visible through it [17]. Typically, this tissue is plentiful and plays a role in determining the shape and size of a gland.

Calcifications are a kind of abnormality that may be noticed on mammography pictures and are one of the most common. Calcification is the term used to describe the presence of calcium in breast tissue [18]. The presence of calcification does not always imply the presence of breast cancer, nor does it always constitute a warning indicator. However, calcification may be a very crucial indicator of cancer in its early stages, which raises the likelihood of successful treatment if discovered in time. There are two kinds of calcification: microcalcification and microcalcification [19]. Microcalcification is characterized by a large quantity of calcium and is an asymptomatic sign of benign calcification, while microcalcification is characterized by a very little amount of calcium, which is less than 0.5 mm and is suggestive of malignant calcification [20].

It is time-consuming and difficult work to manually recognize these histological pictures for the diagnosis of bosom malignant development, and the result may be impacted by the pathologist's knowledge and experience [21]. A consequence of this is that programed inquiry, also known as a computer-assisted examination of histopathological pictures, is increasingly significant in the early diagnosis and detection of breast cancer [22]. However, technological developments in hardware for the programmed localization and evaluation of bosom malignant growth are being delayed by a range of difficulties [23]. To begin with, histopathological pictures of breast disease are high-resolution, fine-grained images with an extremely intricate design that is quite difficult to create [24]. Second, extensive stockpiling is necessary in order to prepare for the histopathological photos that will be taken. Among the challenges to consider is creating appropriate algorithms and models for emphasizing choice, data theft and protection, and other related matters [25]. The higher false-positive rates in breast mammograms are an important test of the effectiveness of adopting the PC-supported framework for bump recognition. If a false-positive test result is not corrected, it might entail prolonged stress, extra radiation exposure, greater medical care costs, and further inquiry [26].

The article "A Breast Cancer Image Classification Algorithm with 2c Multiclass Support Vector Machine" was published in 2023. Journal: J Healthc Eng.

The recurrence of computerized mammogram images provides an opportunity to address the difficult issue of early detection of bosom disease by using profound learning techniques, as demonstrated in the study mentioned above [27].

There are substantial disparities in the states of the bosom tissues according to the writing, and as a result, the benchmarks may be eliminated throughout the screening encounter. In addition to the ROI's size and shape, the morphology of microcalcifications (which is defined by the distance between each little calcification) is a significant feature to consider when defining the ROI [28]. In contrast to a fixed-scale strategy, which is based on the distance between single calcifications used to describe the microcalcification bunch, an invariant-scale strategy is a novel technique that predicts the different morphological angles for the radiologist. Histogram-based methodologies and the computation of optimum edges, in addition to mass division and layout, are a professional approach to calcification and calcification [29].

In general, classification is the last step of medical image processing procedures, during which each and every unidentified pattern is assigned to a category and assigned to a label. The classification job is completed in two steps, which are the training stage and the testing stage. When predicting the labels of classes, a training data set is utilized as a predictor in the training step [30]. With the aid of the trained classifier, photos are reviewed to see whether they belong to a malignant image or a noncancerous image during the testing stage. If they do not, the images are discarded. A total of seven different classifiers are employed in this study, namely, the Support Vector Machine (SVM), K Nearest Neighbors (KNN), Naive Bayes (NB), Linear Discriminant Analysis (LDA), Multilayer Perception Neural Network (MLPNN), Random Forest Tree (RFT), and Least Square Support Vector Machine (LS-SVM).

The article "A Breast Cancer Image Classification Algorithm with 2c Multiclass Support Vector Machine" was published in 2023. Journal: J Healthc Eng.

A variety of performance indicators, such as the confusion matrix, the TP, the TN, the FP, the FN, the ROC curve, the sensitivity, the specificity, the precision, the F-measure, the error rate, and the classification accuracy, are often used to assess the proposed CAD system's performance.

The analysis of medical pictures, particularly breast cancer mammography images, is very time-consuming and difficult for a variety of reasons.

Because of the high levels of noise and background information in mammogram pictures, they are not perfectly segregated.

Because of the concealed nature of the breast tissues and the density of the breast tissues, it is difficult to detect lesions.

## 2. Related Works

In this paper, Neslihan Bayramoglu et al. [30], as well as their colleagues, provided the existence of bosom malignant growth, which is the most frequent illness among women and can only be determined by microscopic inspection of breast tissues. It is necessary to do a painstaking inspection of tissue pictures at different amplification levels in order to identify clinical assessment bits of information that will result in the proper conclusions throughout the pathology evaluation process. Computerized imaging technologies have advanced to the point where pathology pictures may now be examined using PC vision and artificial intelligence approaches, which have the ability to automate a part of the duties involved in the analytic pathology work process. This type of robotization has the potential to succeed when it comes to taking measurements quickly and precisely, eliminating eyewitness discrepancies, and boosting impartiality [31]. In this research, we suggest the use of convolutional neural networks to characterize breast malignant growth histopathology pictures that have not been amplified, rather than using traditional methods such as contrast enhancement [29]. For a single assignment, we have two different architectures to choose from. CNN is used to anticipating danger and doing many tasks at the same time. CNN has become used for predicting both potential damage and the extent of visual amplification [28]. It is necessary to utilize the British dataset in order to conduct assessments and establish connections with prior results. According to the results of the tests, our free CNN approach boosts the display of the amplification explicit model [27].

The article "A Breast Cancer Image Classification Algorithm with 2c Multiclass Support Vector Machine" was published in 2023. Journal: J Healthc Eng.

Ross Girshick Donohue [2] delivered a presentation. According to the highly regarded PASCAL VOC dataset, the rate of object recognition execution has slowed significantly in recent years. Arrhythmic collection frameworks, which often combine a lot of low-level picture features with large-level settings, are the most successful strategies when it comes to collecting information randomly [26]. As a consequence of this research, we have developed a simple and adaptable location calculation that improves mean normal exactness by more than 30% as compared to the previous best result in VOC 2012—achieving a mean average precision (mAP) of 53.3 percent. In our methodology, we combine two key pieces of knowledge: (1) when marked preparation information is scarce, administering prepreparing for an assistant assignment, followed by space explicit adjusting, results in critical presentation support; and (2) when marked preparation information is scarce, administering prepreparing for an assistant assignment, followed by space explicit adjusting, results in critical presentation support [25]. We refer to our approach as R-CNN (regions with CNN). Due to the fact that we mix regional suggestions with CNNs, we have [3] highlights. In addition, we compared R-CNN to OverFeat, a newly suggested sliding-window finder based on a similar CNN approach that was just presented [24].

They published their results in which Noura et al. [4] were all involved. The half-and-half deeper neural organization of the Markov model, compared to the standard Gaussian blend model-HMM, seems to greatly boost the execution of discourse acknowledgment sentences. As a result of its capacity to demonstrate extensive links in discussion highlights, the DNN has had a role in the exhibition's development to some extent. In this study, we show that employing convolutional neural networks may result in an even higher error rate decrease. Starting with a quick explanation of the core CNN and how it may be utilized for voice recognition, we go on to more advanced topics [23]. As an alternative, we propose a restricted weight-sharing method that will allow us to more readily present discussion highlights [22]. A degree of invariance in CNNs is shown through neighborhood networks, weight sharing, and pooling, which are all sensitive to minor variations in discourse highlights along the recurrent hub, which is critical for managing speaker and climate fluctuations [21]. According to the results of the TIMIT telephone acknowledgment and voice search huge jargon discourse acknowledgment projects, CNNs have a (6–10) percent reduction in mistake rates when compared to deep neural networks (DNNs) [20]. As a whole, it can be said that artificial neural networks have benefited from the use of “profound” learning, a term that refers to the number of hidden layers in the neural organization as well as the dynamics and, according to some records, mental believability of depictions acquired in the layers farthest removed from information [19]. A review of approaches suggested for evaluating bosom malignant development histopathological pictures is provided by Veta et al. in [5].

The article "A Breast Cancer Image Classification Algorithm with 2c Multiclass Support Vector Machine" was published in 2023. Journal: J Healthc Eng.

This examination field has become increasingly important since the introduction of slide imaging scanners, which are capable of performing proficient and high-throughput put histopathology slide digitalization and are gradually replacing the optical magnifying instrument as the primary tool used by pathologists [18]. Breast cancer is the most frequent kind of tumor among women, and image inspection methodologies that are focused on this illness have a significant potential to minimize the workload in a conventional pathology lab while simultaneously improving the quality of their interpretation [17]. This paper is purportedly designed to be used as a presentation for those who are not technical specialists. Beginning with an overview of the tissue planning, staining, and slide digitization operations, it moves on to a discussion of the various image handling techniques and applications, which include everything from tissue staining inquiry to PC-supported findings and anticipating breast cancer patients [16].

## 3. Proposed System

I proposed two approaches for categorizing bosom disease histology pictures into safe and dangerous subclasses based on their morphological characteristics. The first methodology is based on the extraction of a collection of handmade highlights encoded by two coding models and generated by assist vector machines, whereas the second methodology is based on the design of Convolutional neural networks. The second methodology is based on the extraction of a collection of handmade highlights encoded by two coding models and generated by assist vector machines. In this paper, a robotized framework for bosom malignant development mammography pictures was presented for the first time, and it made use of a Multisupport Vector Machine and a deep learning instrument. The preplanning stage is straightforward, and it is distinguished by the use of noise, as well as the completion of cleaning and resizing operations. Using the Microsoft Visual Studio Visualization Module, the prepared organization collects, extracts, and groups images. Multiple Support Vector Machines (MSVMs) are utilized to produce better results than a decision tree model. There are DL beat cutting-edge tactics such as the MLP and the J48 + K-mean grouping WEKA methodology, according to the quantitative analysis and clearance. A 2 percent improvement in exactness was seen across the board. The major purpose of this experiment was to examine the consistency of arrangement exactness when bigger datasets were used, which was accomplished via the expansion of the datasets. Eventually, it is hoped that deep learning internal layers would be able to cope with the huge breadth of the deep learning organization and assist radiologists in approving large datasets in less time.

The article "A Breast Cancer Image Classification Algorithm with 2c Multiclass Support Vector Machine" was published in 2023. Journal: J Healthc Eng.

In order to achieve effective diagnosis and classification of breast cancer, the feature extraction step is very critical. Since then, the feature extraction approaches have helped to increase the overall performance of the CAD system in question. There are three basic approaches for feature creation and extraction described in this section: wavelet decomposition, curvelet decomposition, and shearlet decomposition, which will be covered further in this section. The first section of this section describes the implementation of CAD for the early detection and classification of breast cancer tissue using DWT, DCT, and DST with an SVM classifier in the context of breast cancer tissue. The second section of this section describes how to identify and classify microcalcification lesions using an SVM classifier and DST, as well as how to treat them. In this study, the suggested system takes into account a number of strategies that have been employed by earlier researchers that are relevant to the thesis work and incorporates them. In order to improve classification accuracy, new strategies have been developed that are based on the concepts discussed in this section, among other things. This section provides a full overview of feature extraction methods and numerous transformations, followed by an explanation of the approach that has been provided in the previous section. Through the course of this thesis study, statistical texture characteristics of the first and second orders are discovered and retrieved.

The training phase and the testing phase are the two primary stages of this research project, which are carried out in parallel. During the training phase, classifiers for the proposed CAD are trained in such a manner that they can distinguish between normal and abnormal pictures by comparing them to specified normal and abnormal images.

The article "A Breast Cancer Image Classification Algorithm with 2c Multiclass Support Vector Machine" was published in 2023. Journal: J Healthc Eng.

### 3.1. Architecture Diagram

Figure 1 represents the architecture of the proposed work. Picture segmentation is the process of dividing a single image into many segments or areas, each of which is visually coherent. The process of dividing an image into distinct areas or segments in such a way that each region is homogenous and makes it simpler to study the picture is described as follows. Image segmentation is defined as follows. To do this, the purpose of segmentation is to locate and identify the required portion of a picture that has more information about particular facts than any other portion of the image. The outcome is that particular regions of interest are separated from the real picture in order to distinguish certain areas within the image and also to assist radiologists in their diagnosis of the image. Image segmentation is extensively employed in a variety of applications such as remote sensing and medical imaging. Radiologists employ breast pictures with regions of focus to look for abnormalities such as microcalcifications (both benign and malignant), masses, and other growths (benign and malignant).

It is quite difficult to automate the identification of areas of interest. Consequently, in this study effort, the ROI picture is manually cropped using an abnormality location, which is accessible in the MIAS database.

#### 3.1.1. Flowchart

In image transformation, the goal is to collect spatial frequency information, which will be utilized as an input to the feature extraction phase later in the process. The image transformation approach is used in medical image processing and pattern identification since it reduces the dimensionality of the picture. Through the use of the compression approach, this dimensionality reduction may be accomplished. There are three distinct transformations that are employed in this thesis, notably the wavelet transform, the curvelet transform, and the shearlet transform, among others. Feature extraction is a critical component of CAD performance since it determines how well the system performs. In certain circles, feature extraction is referred to as “description.” When it comes to description, it is the process of extracting qualities that provide some quantitative information of importance in order to distinguish one class of items from another class of objects. When the input data to be manipulated is complicated, it is first translated into a collection of features known as a feature vector before being utilized. It is the process of gathering information about images such as color, shape, and texture, among other things. The features of an image include the relevant information about the picture, and they are employed in the image processing operation (e.g., searching, retrieval, storing).

The article "A Breast Cancer Image Classification Algorithm with 2c Multiclass Support Vector Machine" was published in 2023. Journal: J Healthc Eng.

Figure 2 represents the flowchart of the proposed work. Occasionally, the initial feature set includes information that is both redundant and irrelevant. Feature selection is required in order to locate a subset of relevant characteristics by removing duplicate and irrelevant features from the collection of available features. As a result, the categorization accuracy improves significantly. The techniques of feature selection include feature ranking and subset selection, which are both sorts of feature selection methods. In this thesis work, GA is used to choose feature subsets from a large number of candidates. In general, classification is the last step of medical image processing procedures, during which each and every unidentified pattern is assigned to a category and assigned to a label. The classification job is completed in two steps, which are the training stage and the testing stage. When predicting the labels of classes, a training data set is utilized as a predictor in the training step. With the aid of the trained classifier, photos are reviewed to see whether they belong to a malignant image or a noncancerous image during the testing stage. If they do not, the images are discarded. A total of seven different classifiers are employed in this study, namely, the Support Vector Machine (SVM), K Nearest Neighbors (KNN), Naive Bayes (NB), Linear Discriminant Analysis (LDA), Multilayer Perception Neural Network (MLPNN), Random Forest Tree (RFT), and Least Square Support Vector Machine (LS-SVM).

### 3.2. Proposed Process Explanation

#### 3.2.1. Breast Cancer Screening

The primary problems of breast illness are vague, but they disclose true entanglements based on the patients' sexual orientation, age, and genetic history. Because of its tiny size, the placement of the bosom tumor is curable, and it can improve patient observation. Furthermore, competent judgment and appraisal of bosom malignant growth based on bosom thickness aid doctors in the detection of masses and calcification.

#### 3.2.2. Breast Cancer Is on the Rise

A breast mass is a cluster of tissues implicated in damage that is considered an unambiguous marker of breast cancer progression. Depending on its morphological construction, such as thickness, shape, and edge features, mass can be hazardous or useful. The ROI division measurement is affected by the mass's form and size. Kind-hearted masses are frequently seen in oval, lobular, and circular shapes with smooth limits, but destructive masses have unpredictable edges with poorly determined estimated margins. Depending on the size and state of the majority, the radiologist may recommend additional breast examinations. Based on mass size and shape, it created a mass division approach to detect ROI and bosom anomalies.

The article "A Breast Cancer Image Classification Algorithm with 2c Multiclass Support Vector Machine" was published in 2023. Journal: J Healthc Eng.

#### 3.2.3. Image Preprocessing

An image has a number of extra pixels that are not used to represent any data about the picture. This preplanning is predicted to reduce the organization's computational intricacy and overhead, allowing us to increase results. The initial unbiased prehandling is the preprogrammed trimming of the mammograms' bosom area. To create this balance, photos having a bosom on the other side were flipped to an areola, emphasizing the right side. At that moment, the path toward editing is. To remove data from the foundation, such as names and wedges in the images, the dark scale image is the first threshold into a double image, and then morphological tasks are done to the paired image to remove all undesirable small articles. A variety of methods and calculations are commonly used to address this overall classification as a starting point for edge location and district marking, and changes to these strategies, locale naming, and examinations are almost direct calculations that have been utilized for quite some time to segregate, measure, and build up potential areas.

After the successful extraction of ROI, DST is applied to the ROI image for the purpose of feature construction. DST transforms the ROI image into a collection of subbands of the same size. The number of subbands produced depends upon the number of levels and number of directions, which is used to decompose the images. In this work, the images are decomposed using different levels and different directions. The decomposition levels vary from 2 to 5 and the direction varies from 2 to 64. The output of the decomposition process is nothing but the generation of shearlet coefficients. From these coefficients, specific features are extracted. In this approach also, the same, four first-order statistical features, namely, mean, variance, skewness, and kurtosis, are extracted from the shearlet coefficients. These features are fused to form the feature vectors and it is used as one of the inputs for the classification purpose. Classification is the important and critical step in medical image analysis, in which each unknown pattern is assigned to a particular category. The classification task is done based on two stages, namely, training and testing stages. In the training stage, a training data set is used to predict the labels of a class. In the testing stage, the testing image is checked whether the given testing mammogram is a cancerous or noncancerous one by using the trained classifier. In this stage, the SVM classifier is considered for the classification task. Here, classification is done in two steps. In step 1, an unknown mammogram image is classified as either cancerous or noncancerous.

The article "A Breast Cancer Image Classification Algorithm with 2c Multiclass Support Vector Machine" was published in 2023. Journal: J Healthc Eng.

#### 3.2.4. Image Capture

Procure/acquire the report's image in shading, dark level, or twofold organization. Many remarks on images are required for the improvement of a productive DL model, which is difficult to meet essentially, for example, physically splitting and identifying the image, information upgrade, and prehandling demands for executions. Initially, the mammography was converted to a versatile dark arrangement that does not contaminate the information when it is packaged. The actual image has no name and no meaning. Until it is used, it should be physically separated and identified. However, photographs taken in real life frequently have flaws that influence the nature of the element extraction.

#### 3.2.5. Binarization

It converts the received image to a paired configuration with the purpose of finding an edge that separates the foreground and foundation data. The determination of a reasonable limit is typically an experimental interaction. A dark degree of 128 is set on the edge. This is especially problematic when the distinction between text pixels and the foundation is low.

#### 3.2.6. Noise Reduction

During the information extraction process, binarization of pictures is commonly required, which removes the majority of the turbulence and replaces each pixel in the picture, the character, and the pixel behind the scenes with double 0 and 1 values that are independent of one another. Following binarization, it is common practice to filter reported pictures in order to decrease noise. To reduce agitation or to repair the borders of the characters, smoothing activities are used in twofold archival images. These activities include filling tiny holes or eliminating minor knocks from the edges of the characters' faces, among other things. It is essential that sifting be capable of smoothing and eliminating disturbance. A local activity in which the estimation of any random pixel in the producing image is dictated by applying some computation to the estimates of the pixels in the immediate neighborhood of the corresponding input pixel is referred to as “separating.” To keep noise levels as low as possible, a variety of measures are used.

#### 3.2.7. Thresholding Process

Thresholding is the simplest basic technique for image splitting. Thresholding can be used to create paired images from a low-resolution image. Parallel images are formed by dividing shading images. The division is in the process of assigning each pixel in the source image to at least two classes. If there are numerous classes, the typical result is a few parallel images. Thresholding is used in image preparation to divide a picture into smaller pieces or to remove them entirely, utilizing at least one tone or dim scale worth characterizing their limit. The benefit of acquiring an initial double picture is that it minimizes the complexity of the information and improves the cycle of acknowledgment and characterization.

The article "A Breast Cancer Image Classification Algorithm with 2c Multiclass Support Vector Machine" was published in 2023. Journal: J Healthc Eng.

Figure 3 represents the region growth of the proposed work. Due to the large number of possible options, selecting the most appropriate hyperplane is a tough undertaking. There is just a slight separation between the classes between the hyperplanes “a” and “c”. Classifications are separated by the hyperplane “b,” which has the largest margin. To this end, a Support Vector Machine (SVM) classifier is trained in such a manner that it can identify the hyperplane that divides various classifications and where the margin between the two classes is at its largest. Support vectors are identified by the SVM classifier as data points that are close to the ideal separation hyperplane, which are then classified. The margin of the SVM classifier is defined as the distance between the separating hyperplane and the closest of the positive and negative data points.

Baker (1982) defined SVM as a binary linear classifier that accomplishes classification by generating hyperplanes in a multidimensional space that segregate the instances with distinct class labels. SVM is basically a nonprobabilistic binary linear classifier. SVM utilizes an iterative training procedure to generate an ideal hyperplane, which is utilized to minimize an error function in order to do this.

#### 3.2.8. Image Segmentation

Picture division is the cycle that divides a picture into its basic components or elements. The extent to which this development is done depends on the issue being addressed; i.e., the division should stop when the objects of interest in an application have been confined, e.g., to self-governing air-to-ground target security, assuming our advantage lies in distinguishing vehicles on a street. Picture thresholding algorithms are used for image division.

#### 3.2.9. Convolutional Neural Network

Figure 4 represents the Convolutional architecture. The convolutional neural organization is a deep learning calculation that is often used for image arrangement, highlight extraction, object finding, and face recognition, among other things. CNN begins with randomly defined loads and then changes these loads after each layer. CNN will use these loads to forecast the outcome of the approval and testing procedures after the model has been built. CNN is being used more and more for image division and clinical image processing. As a result, the CNN model incorporates features from back-proliferation by applying multiple layers including convolution, pooling, and totally connected layers. CNN's development is divided into two stages. In the first stage, pixels are convolved with a piece or channel, providing the convolution of the picture square and the part. The profundity of the channel will be the same as the profundity of the information, and its stature and width will be determined by the size of the organization. The second most significant development is pooling or subexamining, which can be of many forms, such as max pooling, min pooling, and average pooling. Overfitting and dimensionality are reduced by using CNN's pooling layer. Often, odd channels are used for pooling activities by the client in the pooling layer.

The article "A Breast Cancer Image Classification Algorithm with 2c Multiclass Support Vector Machine" was published in 2023. Journal: J Healthc Eng.

### 3.3. Algorithm of Canonical Correlation

Canonical Correlation Analysis is a well-known approach in multivariate measurable examination that has been widely used in financial aspects, meteorology, and a variety of sophisticated data preparing sectors, for example, correspondence hypothesis, factual sign handling, and Blind Source Separation. CCA was developed as a method of assessing the direct relationship between two multidimensional arrangements of elements and was then extended to a few data collections. CCA is typically generated as a summed up Eigen esteem issue. However, due to their high computational expense, the immediate application of Eigen deterioration procedures is frequently unsuitable for high-dimensional informational indexes as well as for varied situations.

### 3.4. 2C Algorithm Using in Proposed System

Canonical correlation analysis (CCA) is a subspace learning approach that seeks to learn a common feature space by observing cross-domain data pairings and maximizing the correlation between the projected cross-domain data pairs. CCA's capacity to link diverse cross-domain data is a significant advantage (i.e., source and target domain data in different feature representations). CCA has been used successfully to handle a number of cross-domain visual classification tasks, including the PRID. Several CCA versions have been developed, including the Ranking CCA for learning query and picture similarities, which learns a bilinear query picture similarity function while also adjusting the subspace to retain the preference relations. The tensor canonical correlation analysis maximizes the canonical correlation of several viewpoints at the same time.

Figure 5 represents the 2C algorithm of the proposed work. This section provides an overview of canonical correlation analysis (CCA) and constrained CCA. The purpose of this study is to discover a link between the two sets of variables. CCA, as the name implies, quantifies the link between two sets of variables by using correlation coefficients. The term &quote; canonical & quote; refers to the coordinate system used to calculate the correlation.

The article "A Breast Cancer Image Classification Algorithm with 2c Multiclass Support Vector Machine" was published in 2023. Journal: J Healthc Eng.

#### 3.4.1. Support Vector Machine

The Support Vector Machine was first proposed and has subsequently generated significant money in the AI research field. A few recent investigations have indicated that, on average, assist vector machine scans transmit more information in terms of arrangement precision than other information grouping calculations. SVM is a twofold classifier that is dependent on regulated realization and provides superior performance over other classifiers. By generating a hyperplane in high-dimensional element space that may be used for grouping, SVM establishes an order between two classes.

#### 3.4.2. Extraction of Characteristics

Feature extraction is a method for extracting noteworthy highlights from an input image. We extract deteriorating tissue from the portioned image with the presence of insignificant meaningless components in the examination, and it resolves dimensionality loss. Separating useful data for volume calculations is a huge undertaking. Separating the highlights from the photos is a huge step forward in photo grouping. Highlights are made locally in the standard picture order process using some specific guidelines and procedures. However, cutting-edge convolutional neural network approaches for the most part extract the highlights universally utilizing parts, and these global features have been used for image arrangement.

Figure 6 represents the tissue classification of the proposed work. Tissues are classified as normal or pathological during the tissue arrangement procedure. The arrangement is carried out by starting with the more discriminative highlights and gradually adding less discriminative highlights until grouping execution is no longer improved. For this purpose, many characterization methods such as SVM, artificial neural organization, and k Nearest Neighbor are used.

## 4. Results and Analysis

The MIAS database is being utilized for experimental purposes in this investigation. There are 322 breast photos in all, divided into the categories of normal, microcalcification, mass, benign, and malignant. All of the photos have a resolution of 1024 by 1024 pixels and an accuracy of 8 bits (gray level). In addition, the database provides information regarding the locations of anomalous events. A region of interest (ROI) picture of size 256 × 256 pixels is extracted from the source image based on the locations of anomalies. A total of 70 photographs are obtained for normal instances, while 25 microcalcification images (13 benign and 12 malignant images) are taken for abnormal cases. The images are used for assessment purposes. Figures 7(a)–7(d) represent the result comparison.

The article "A Breast Cancer Image Classification Algorithm with 2c Multiclass Support Vector Machine" was published in 2023. Journal: J Healthc Eng.

The graphic depicts the evaluation of applied filters and the calculation of three image quality metrics such as PSNR, SNR, and MSE for three different kinds of mammography pictures. The fatty group of benign mammography pictures had the greatest SNR value. The SNR has a value of 21.38. When compared to the other categories of mammography pictures, this is the highest value shown in Table 1. In terms of PSNR value, the malignant category of the fatty mammography picture has attained the highest value when compared to the other mammography picture categories. In terms of MSE, the applied filter produces moderate error values when compared to the other salt and pepper noise filters. The applied filter has the lowest MSE value of 52.91. When compared to other types of mammography pictures, the MSE values appear to be high.

Figure 8 gives the graphical analysis of the proposed work. Comparison of two algorithms and chart.

All approaches are compared based on the accuracy of cancer segmentation, comparison of findings based on statistical values, and visual comparison of breast cancer images. The accuracy of the segmentation approach is determined by comparing it to a manually segmented ground truth image in Table 2. The area of impacted cancer is considered as a measure of the performance of the compared two algorithms, and the algorithm may be compared with a segmented value by physicians by using the area of impacted cancer as a parameter of measurement.

Figure 9 represents the comparison graph of the proposed work. The comparison table shows that the suggested 2C algorithm with MSVM outperforms a decision tree model in terms of accuracy.

Figure 10 represents the error rate and graphical representation of the proposed work. Testing and evaluation measures such as TP, FP, TN, FN, sensitivity, specificity, precision, F-measure (error rate), ROC curve (receiver operating characteristic curve), and classification accuracy are used to evaluate the produced system. TP is the number of normal images that have been appropriately categorized as noncancerous images. TN is the number of aberrant images that have been accurately diagnosed as malignant images. FP is the number of normal photos that have been incorrectly labeled as malignant images. FN is the number of abnormal pictures that have been incorrectly categorized as noncancerous. Sensitivity is often referred to as the True Positive Rate or Recall Rate (TPR). This is defined as the proportion of pictures with abnormalities whose output is positive, and it is determined using the following formula:

(1) $$\begin{array}{c} \text{sensitivity}=\frac{\text{TP}}{\left(\text{TP}+\text{FN}\right)}. \end{array}$$

Specificity is defined as the percentage of images with normal, whose ut is negative and it is calculated using the following equation:

(2) $$\begin{array}{c} \text{specificity}=\frac{\text{TN}}{\left(\text{TN}+\text{FP}\right)}. \end{array}$$

Classification accuracy is defined as the number of correctly divided ages, which is divided by the total number of implied images and then by 100 to turn it into a percentage. It is calculated using the following equation:

(3) $$\begin{array}{c} \text{classification accuracy}=\frac{\left(\text{TP}+\text{TN}\right)}{\left(\text{TP}+\text{FP}+\text{TN}+\text{FN}\right)}. \end{array}$$

Precision is defined as the number of true positives, which is led by the number of true positives and false positives and it is calculated as

(4) $$\begin{array}{c} \text{precision}=\frac{\text{TP}}{\left(\text{TP}+\text{FP}\right)}. \end{array}$$

False-Positive Rate (FPR) is defined as the number of false motives, which is divided by the number of false positives and true negatives; it is calculated

(5) $$\begin{array}{c} \text{FPR}=\frac{\text{FP}}{\left(\text{FP}+\text{TN}\right)}. \end{array}$$

The F-measure or F-score is a precision recall. The F-measure is determined by using

(6) $$\begin{array}{c} F-\text{measure}=2*\text{Recall}*\frac{\text{Precision}}{\text{Recall}+\text{Precision}}. \end{array}$$

SVM classifier has higher classification accuracy than the other classifiers, as shown by the results of the experiment. As a result of the regularisation parameter in the SVM classifier, it achieves higher classification accuracy and prevents overfitting of the model. It is resistant to noise and, more importantly, it takes advantage of the kernel technique.

The article "A Breast Cancer Image Classification Algorithm with 2c Multiclass Support Vector Machine" was published in 2023. Journal: J Healthc Eng.

Figure 11 represented the error rate calculation.

## 5. Conclusion

Breast cancer is a real threat to women all over the world, and it is a major cause of female mortality. Improving present breast disease conditions is a big problem, and it can be addressed by adequate assessment, discovering and fitting patients, and clinical administration. A standard check of the disease and distinguishing evidence of bosom malignant growth in the earlier stages can save many lives. The issue with cancer evolves throughout time, as the appearance, appropriation, and primary math of the cells alter over time due to the compound alterations that occur inside the cell. The changing structure of cells can be distinguished by examining biological images obtained from mammography, MRI, and other methods. For the first time, a robotized framework that employs a Multisupport Vector Machine and a deep learning instrument for breast cancer mammography images was proposed. The preplanning step is straightforward, with commotion, handling, and resizing tasks. The prepared organization handles acquired images for highlight extraction, and the order is completed by applying MSVM. When compared to a decision tree model, a crossover method of K-mean bunching and MSVM produces better results. The quantitative study and approval confirm that the proposed DL method outperformed the best-in-class procedures, namely, MLP and the J48+K-mean grouping WEKA strategy. In general, there was a 2% improvement in exactness. The primary goal of this investigation was to test the constancy of characterization precision when given larger datasets, which were therefore expanded. The long-term goal is to deal with the massive breadth of the organization of deep learning internal layers and aid radiologists in approving massive datasets in less time.

This paper also describes the training approach and testing method that are utilized for the identification of microcalcification utilizing DST and a linear SVM classifier, which are both discussed in detail in Section 2. With the SVM classifier, this proposed study produces a classification accuracy of 99.28 percent for the normal/abnormal case of microcalcification during the first step of the classification process and a classification accuracy of 100 percent for the benign/malignant case of abnormal microcalcification detection during the second step of the classification process. Furthermore, the performance of this work is compared to that of previously published research work, and it demonstrates the increase in accuracy of the suggested work when compared to that of other previously published techniques, which is a significant benefit. Consequently, in Section 4, DST is used to deconstruct mammography pictures, and then, the different statistical texture characteristics are recovered from the decomposed images in Section 5. This section describes the CAD approach for breast cancer diagnosis, which includes the use of several classifiers in addition to the SVM classifier and the DST.

## Figures and Tables

**Figure 1:** Architecture.

**Figure 2:** Flow process.

**Figure 3:** Region growth process.

**Figure 4:** Convolutional neural network structure.

**Figure 5:** 2C algorithm process.

**Figure 6:** Tissue classification process.

The article "A Breast Cancer Image Classification Algorithm with 2c Multiclass Support Vector Machine" was published in 2023. Journal: J Healthc Eng.

**Figure 7:** (a–d) Segmented results of the proposed work.

**Figure 8:** An accuracy rate comparison.

**Figure 9:** Comparison graph.

**Figure 10:** Training data epoch.

**Figure 11:** Error rate calculation.

**Table 1:** Table of the comparison graph.

Abnormality status	Background tissue	SNR (in ratio)	PSNR (in ratio)	MSE (in average)
Normal	Fatty	20.067	28.485	92.167
	Fatty glandular	18.780	28.936	83.073
	Dense glandular	19.872	28.408	93.798

Benign	Fatty	21.382	29.957	65.672
	Fatty glandular	19.626	26.923	132.050
	Dense glandular	18.348	27.404	118.212

Malignant	Fatty	21.080	39.895	52.913
	Fatty glandular	21.142	29.022	81.433
	Dense glandular	20.886	29.525	72.528

**Table 2:** Comparison of two algorithms and chart.

Algorithm	Accuracy	Sensitivity	PSNR
2C algorithm	98.64	88.49	77.74
Multiclass support vector machine	95.56	95.49	63.26

## Data Availability

The data that support the findings of this study are available on request from the corresponding author.
